# MiR-19a suppresses ferroptosis of colorectal cancer cells by targeting IREB2

**DOI:** 10.1080/21655979.2022.2054194

**Published:** 2022-05-21

**Authors:** Hongwei Fan, Rong Ai, Suen Mu, Xuemin Niu, Zhengrong Guo, Lin Liu

**Affiliations:** a Department of Gastroenterology, Shijiazhuang People’s Hospital, Shijiazhuang, Hebei, China; b Department of Pathology, Shijiazhuang People’s Hospital, Shijiazhuang, Hebei, China

**Keywords:** miRNA, colorectal cancer, ferroptosis, miR-19a, iron-responsive element-binding protein 2, cell proliferation

## Abstract

Colorectal cancer (CRC) is the most common malignant tumor occurred in digestive system. However, the prognosis of CRC patients is poor. Therefore, it is urgent to illuminate the mechanism suppressing CRC and explore novel targets or therapies for CRC treatment. MicroRNAs (miRNAs) are a class of non-coding RNAs with a length of 20–23 nucleotides encoded by endogenous genes, which are associated with the development of a variety of cancers, including CRC. Studies have shown that miR-19a is identified as oncogenic miRNA and promotes the proliferation, migration and invasion of CRC cells. However, the relationship between miR-19a and ferroptosis in CRC remains unknown. Here, we reported that iron-responsive element-binding protein 2 (IREB2), as an inducer of ferroptosis, was negatively regulated by miR-19a. IREB2 is a direct target of miR-19a. In addition, ferroptosis was suppressed by miR-19a through inhibiting IREB2. Thus, we proposed a novel mechanism of ferroptosis mediated by miR-19a in CRC cells, which could give rise to a new strategy for the therapy of CRC.

## Highlights

- This study demonstrated that IREB2 was the target of miR-19a in CRC for the first time.
- This study revealed that miR-19a suppressed ferroptosis in CRC through inhibiting IREB2 expression for the first time.
- MiR-19a might be a novel therapeutic target for CRC treatment.

## 1. Introduction

Colorectal cancer (CRC) is the most common malignant tumor occurred in digestive system and a leading cause of cancer-related death in the world [1,2]. To date, surgical resection is still the major therapy for CRC [3]. However, the prognosis of CRC patients is poor [4]. Therefore, it is urgent to illuminate the mechanism suppressing CRC and explore novel targets or therapies for CRC treatment [5,6].

MicroRNAs (miRNAs) are a kind of small (19–23 nucleotides) non-coding RNA molecules that function as endogenous suppressors of gene expression by binding to the 3’-untranslated region (3’-UTR) of target mRNAs to facilitate translational inhibition or mRNA cleavage [7]. Generally, miRNAs, as crucial post-transcriptional regulators, are involved in many physiological and pathological processes, including autophagy [8,9], cell differentiation [10], cell proliferation [^11–13^], DNA damage and repair [14], organ development [15,16] and tumorigenesis [17,18]. Numerous miRNAs are directly or indirectly correlated with oncogenes and function as oncomiRNAs or tumor suppressor miRNAs, especially in colorectal cancer [17,19,20].

During CRC development, numerous genes have an effect on CRC cell growth, migration, and invasion, including miRNA [^21–23^]. MiR-19a is one of the most important miRNAs and has been reported to be remarkably overexpression in CRC [11,24,25]. miR-19a can also promote the invasion and metastasis of CRC cells via targeting TG2 [26]. In addition, the IREB2 gene belongs to a group of genes that regulate iron homeostasis in mammals. IREB2 mainly registers cytosolic iron status through iron-sulfur switching mechanism [27]. However, the molecular mechanism by which miR-19a affects expression of IREB2 is unclear.

Ferroptosis is an iron catalyzed regulatory necrosis that occurs through excessive peroxidation of polyunsaturated fatty acids (PUFAs) [28]. In recent years, ferroptosis has attracted extensive attention, especially considering the down-regulation and silencing of related genes in the occurrence and implementation of necroptosis in cancers [29]. However, the role of miR-19a in ferroptosis of cancer cells is largely unknown. Thus, the relationship between miR-19a and ferroptosis in cancers remains to be studied.

In this study, we provide evidence that IREB2 is a target substrate of miR-19a. IREB2 can interact with and is suppressed by miR-19a directly. Additionally, we demonstrated that miR-19a deficiency decreases cell proliferation and potentiates LDH overflow via up-regulating IREB2 expression. Thus, the present study might provide a novel strategy for the therapy of CRC.

## 2. Materials and methods

### 2.1 Cell culture

Colorectal cancer cell line HT29 was purchased from the Cell Bank of the Chinese Academy of Sciences (Shanghai, China) and was cultured in Dulbecco’s modified Eagle’s medium. All the cell lines were maintained under the manufacturer’s instructions.

### 2.2. RT-qPCR analysis of miRNAs and miRNA targets

Total RNA was extracted using TRIzol reagent (#15,596,026, Invitrogen, CA, USA). A total of 1 µg of RNA was reverse-transcribed using the ImProm-IITM Reverse Transcription System (#A3800, Promega, WI, USA). Quantitative real-time RT-PCR was conducted using SYBR GREEN qPCR Super Mix (#S2024, Invitrogen, CA, USA). A standard amplification protocol was used according to the supplier’s directions. Primers were listed as follows.

IREB2 forward: 5’-GTCTACTTATATCAGATGCC-3’;

IREB2 reverse: 5’-ACTTATTAAAAAGCTTGATAT-3’;

miR-19a forward: 5’-ACACTCCAGCTGGGTGTGCAAATCTATGCAA-3’;

miR-19a reverse: 5’-CTCAACTGGTGTCGTGGA-3’;

18srRNA forward: 5’-CCTGGATACCGCAGCTAGGA-3’;

18srRNA reverse: 5’-GCGGCGCAATACGAATGCCCC-3’;

U6 forward: 5’-CTCGCTTCGGCAGCACA-3’;

U6 reverse: 5’-ACTTATTAAAAAGCTTGATAT-3’.

### 2.3. Western blotting analysis

Western blotting was performed as previously described [30]. The antibodies used were as follows: GPX4 (#bs-3884 R, Bioss, Beijing, China), IREB2 (#bs-4484 R Bioss), GAPDH (#KC-5G5, Aksomics, Shanghai, China), HRP-conjugated secondary antibodies to rabbit (#4050-05, Southern biotech, AL, USA). Original images of WB were provided in Supplementary.

### 2.4. RNA pull-down assay

The RNA pull-down assay was performed as described previously [31]. In this analysis, the wild-type 5’-biotinylated oligos of miR-19a (5’-UGUGCAAAUCUAUGCAAAACUGA-3’) and the mutated 5’-biotinylated oligos of miR-19a (5’-UACAUGGGUCUAUGCAAAACUGA-3’) were synthesized by Invitrogen. The control biotinylated oligos containing random oligos (5’-UUUGUACUACACAAAAGUACUG-3’).

### 2.5. Cell proliferation assay

The cell proliferation was performed as described previously [32]. 1 × 10^4^ cells were seeded into 96-well culture plate in triplicate. The cell proliferation rate and inhibition rate of gene sensitivity were continuously monitored by colorimetric CCK-8 Assay kit (Keygenbio) until 96 hours.

### 2.6. LDH and cytotoxicity test

Culture medium of HT29 cells were collected to detect released LDH level using LDH-Cytotoxicity Colorimetric Assay kit (#K311-400, Biovsion, CA, USA) according to the manufacturer’s instructions. Besides, the absorbance was measured at 490–500 nm. Furthermore, cytotoxicity was calculated using the following formula: (OD sample − OD low control)/(OD high control − OD low control) ×100%.

### 2.7. Dual-luciferase reporter gene analysis

Cells were cotransfected with psi-CHECK2 and miR-19a or miR-19a inhibitor. After 48 h, the expression of luciferase gene was determined and normalized by Dual-Luciferase reporter assays (#E1910, Promega) according to the manufacturer’s protocol. Luminescence was measured using a Synergy2 plate reader GloMax (Promega).

### 2.8. Statistical analysis

The mean of the three experiments was expressed as the mean standard deviation (SD) calculated by STDEV formula. The significance of all data was estimated by Tukey’s multiple-comparison test in the analysis of variance using SigmaStat 3.5 software. When P < 0.05, it was statistically significant.

## 3. Results

CRC is the most common malignant tumor occurred in digestive system. It is urgent to illuminate the mechanism suppressing CRC and explore novel targets or therapies for CRC treatment. Previous studies have shown that miR-19a promotes the proliferation, migration and invasion of CRC cells. However, the relationship between miR-19a and ferroptosis in CRC remains unknown. Thus, the primary aim of this study was to investigate whether miR-19a suppressed ferroptosis in CRC through inhibiting IREB2, which is an inducer of ferroptosis.

### 3.1. Inhibition of miR-19a has no effect on IREB2 mRNA.

IREB2 was an important promoter of ferroptosis. We confirmed that IREB2 was a target of miR-19a by bioinformatical analysis. The prediction showed that 347–353 bp and 1413–1420 bp of IREB2 3UTR were two binding sites interaction with miR-19a (Figure 1(a)). For further confirm how miR-19a regulates the expression of IREB2, HT29 cells were treated with miR-19a inhibitor to silence miR-19a expression. As shown in Figure 1(b,c), no obvious change in the mRNA expression levels of IREB2 was observed in the HT29 cells silencing miR-19a. Besides, the expression of IREB2 protein was up-regulated by miR-19a silence (Figure 1(d)). Taken together, the regulation of miR-19a on IREB2 might occur at the post-transcriptional level.

**Figure 1.** miR-19a inhibits the expression of IREB2 at the translation level. (a) Bioinformatical analysis shows that IREB2 is a target of miR-19a. (B&C) HT29 cells were treated with NC inhibitor or miR-19a inhibitor before harvest, and the mRNA levels of both miR-19a (b) and IREB2 (c) were determined by RT-qPCR. (d) The expression of IREB2 was determined by western blotting in miR-19a inhibitor treatment HT29 cells.

### 3.2. miR-19a interacts with IREB2.

As shown in Figure 1(a), we know that IREB2 is a target of miR-19a via dataset analysis. We hypothesized that miR-19a directly interacts with IREB2. To test this hypothesis, we used miR-19a or mutant miR-19a probe to pull-down IREB2, RT-qPCR and gel analysis depicted that IREB2 could be pulled down by miR-19a, while mutant miR-19a could not pull down IREB2 (Figure 2(a,b)). In conclusion, our data suggest that IREB2 directly interacts with miR-19a.

**Figure 2.** Identification of miR-19a has an interaction with IREB2. (a) RNA-RNA pull down analysis the relationship of IREB2 and miR-19a, and the expression of IREB2 mRNA in different treatment assays were determined by RT-qPCR. (b) Agarose gel electrophoresis analysis in HT29 cells shows the interaction between miR-19a and IREB2.

### 3.3. miR-19a negatively regulates IREB2.

For further determine the relationship of miR-19a mediates IREB2. HT29 cells were treated with miR-19a inhibitor to determine IREB2 promoter activity by dual-luciferase reporter assay. As shown in Figure 3(a), miR-19a significantly decreased the promoter activity of wild-type IREB2, while remarkably potentiated reporter gene luciferase in miR-19a inhibitor treatment HT29 cells. In addition, we constructed three mutant-binding sites of IREB2 3’UTR plasmids, including two single binding sites mutant and a double binding sites mutant. Similar results were obtained in HT29 cells transfected 347–353 bp (Figure 3(b)) or 1413–1420 bp (Figure 3(c)) single binding sites mutant plasmids. There is no apparent effect in mut-IREB2-3 plasmids transfected HT29 cells after treating with miR-19a or its inhibitor (Figure 3(d)). Collectively, our results indicated that miR-19a binds with and negatively regulates IREB2 rely on binding sites.

**Figure 3.** miR-19a negatively regulates IREB2. (a-d) HT29 cells were transfected with indicated plasmids and were treated with miR-19a or miR-19a inhibitor, IREB2 promoter activity was determined by luciferase values. IREB2: wild-type 3’UTR; mut-IREB2-1: 347–353 binding sites mutant of IREB2; mut-IREB2-2: 1413–1420 binding sites mutant of IREB2; mut-IREB2-3: both of 347–353 and 1413–1420 binding sites mutant of IREB2. Error bars represent data from three independent experiments (mean ± SD). * P < 0.05, ** P < 0.01.

### 3.4. miR-19a attenuates ferroptosis of colorectal cancer cells by suppression of IREB2.

IREB2 was a commonly marker that induced cell ferroptosis. We hypothesized that miR-19a could mediate ferrpotosis via IREB2 inhibition in HT29 cells. To test this hypothesis, we assessed the role of miR-19a and IREB2 by investigating the effects of miR-19a inhibitor or IREB2 overexpression on the viability, cytotoxicity and LDH overflow detection in HT29 cells. As expected, miR-19a silence and IREB2 overexpression significantly decreased the proliferation rate of HT29 cells (Figure 4(a,b)). Furthermore, either inhibition of miR-19a or IREB2 overexpression in HT29 cells induced higher inhibition rate compared to those of control cells (Figure 4(c)). These results indicated that miR-19a promoted HT29 cell proliferation, whereas IREB2 suppressed HT29 cell growth.

**Figure 4.** miR-19a attenuates ferroptosis of colorectal cancer cells by suppression of IREB2. (A&B) The cell proliferation in HT29 cells expressing the indicated proteins or treat with indicated inhibitor was tested by the CCK-8 assay. Results presented represent the means of triplicate experiments ± SEM. *P < 0.05, **P < 0.01. (c) Inhibition rates of miR-19a inhibitor and IREB2 gene sensitivity in HT-29 cells, Inhibition rate = (1- mean OD value of the experimental group/mean OD value of the control group) ×100% (same time as cell proliferation). (D&E) HT29 cells were treated as in (a) and LDH overflow detection and related inhibition rate were determined by CCK-8 assay. Results presented represent the means of triplicate experiments ± SEM. * P < 0.05, ** P < 0.01.

In addition, we detected LDH overflow and related cytotoxicity in HT29 cells. Our results showed that HT29 cells treated with miR-19a inhibitor or overexpression of IREB2 remarkably increased LDH overflow compared to the control cells (Figure 4(d)). The cytotoxicity of HT29 cells with the same treatment depicted similar results on cell inhibition rate (Figure 4(e)).

Taken together, our results revealed miR-19a attenuates ferroptosis of colorectal cancer cells via suppressing IREB2.

## 4. Discussion

Ferroptosis was originally a unique form of cell death induced by small molecules, such as erastin, Ras-selective lethal small molecule (RSL)-3, and buthionine sulfoximine, which was used to screen its selective cytotoxicity to cells overexpressing carcinogenic mutant HRAS [33,34]. Morphologically, cell ferroptosis has a typical necrotic morphology, accompanied by abnormal small mitochondria with decreased crista, a condensed membrane, and a ruptured outer membrane [28]. IREB2 (iron response element-binding protein 2) is RNA-binding protein that regulates iron levels through regulating the translation and stability of mRNAs that affect iron homeostasis upon iron depletion [35].

In this work, we demonstrated that IREB2 was a target substrate of miR-19a. IREB2 interacts with and is suppressed by miR-19a directly. Additionally, we demonstrated that miR-19a deficiency decreases cell proliferation and potentiates LDH overflow via up-regulating IREB2 expression. Over the past decade, more direct evidence for iron-dependent ferroptosis comes from the inhibition of IREB2, a master transcription factor of iron metabolism [35]. Suppression of IREB2 expression by RNAi or miRNAs significantly increases iron metabolism-associated gene expression (F-box and leucine-rich repeat protein 5, iron-sulfur cluster assembly enzyme, FTH1, and FTL) [36]. The functional regulatory of IREB2 polymorphism are unclear. The protein product of the IREB2 gene is involved in maintaining human cellular iron balance. It has been reported that smokers had higher concentrations of iron in their lungs [37].

In addition, we also found that miR-19 inhibition induced lethal reactive oxygen species (ROS) production; similarly, IREB2 overexpression also promoted ROS increase. The accumulation of ROS derived from iron metabolism is a common characteristic of ferroptosis [38]. Glutathione peroxidase 4 (GPX4) functions as a negative regulator of ferroptosis by limiting ROS production and reducing cellular iron uptake [39]. In contrast, NADPH oxidase and p53 act as positive regulators of ferroptosis by promoting ROS production, respectively [40]. As a member of miR-17-92 cluster, miR-19a participates not only in the development of organs, such as heart and lung, but also in tumorigenesis, including glioma, bladder cancer, breast cancer, pancreatic cancer, gastric cancer and colorectal cancer (CRC) [24^,41–44^]. Besides, miR-19a also inhibits p53 and PTEN expression in cell proliferation. P53 may also has a key role in relationship of miR-19a and ferroptosis. Furthermore, miR-19a also mediate cancer development, especially in CRC. In addition, we found another new pathway that miR-19a maybe participant in regulating cell proliferation via ferroptosis regulatory by IREB2 inhibition for the first time.

Multiple promotors and suppressors of ferroptosis have been identified. Understanding the molecular mechanisms and signaling pathways of ferroptosis may provide new diagnostic and therapeutic methods to regulate cell proliferation and apoptosis in human disease, especially in colon cancer. In addition to iron-mediated ROS production by Fenton reaction, nicotinamide adenine dinucleotide phosphate (NADPH)-dependent lipid peroxidation and GSH depletion are also important for the induction of ferroptosis [33,45,46]. We found that miR-19a silence by its inhibitor suppresses IREB2 expression and decreases cell growth, thus inhibiting ferroptosis. But how miR-19 mechanical regulatory in ferroptosis in CRC need more depth research. The role of miR-19a in cell ferroptosis still remains further study. Moreover, miR-19a binds with and suppresses IREB2 expression, thus regulating ferroptosis maybe an important regulatory progress in CRC cell growth.

## 5. Conclusions

In summary, this study revealed that IREB2 was negatively regulated by miR-19a in CRC cells. In addition, ferroptosis was suppressed by miR-19a through inhibiting IREB2. Thus, our results proposed a novel mechanism of ferroptosis mediated by miR-19a in CRC cells, which could give rise to a new strategy for the therapy of CRC.

## Supplementary Material

Supplemental Material
